This article has been retracted.

# Chlorogenic Acid Prevents Microglia-Induced Neuronal Apoptosis and Oxidative Stress under Hypoxia-Ischemia Environment by Regulating the MIR497HG/miR-29b-3p/SIRT1 Axis

**DOI:** 10.1155/2022/1194742

**Published:** 2022-05-25

**Authors:** Yong Fan, Yongkun Li, Yongkai Yang, Kunzhe Lin, Qingqiang Lin, Shenghui Luo, Xiaohui Zhou, Qun Lin, Fan Zhang

**Affiliations:** ^1^Central Laboratory, Affiliated Fuzhou First Hospital of Fujian Medical University, No. 190 Dadao Road, Fuzhou 350009, China; ^2^Department of Neurology, Fujian Provincial Hospital, Shengli Clinical Medical College of Fujian Medical University, No.134 East Street, Fuzhou 350001, China; ^3^Neurosurgery Department, Affiliated Fuzhou First Hospital of Fujian Medical University, No.190 Dadao Road, Fuzhou 350009, China; ^4^College of Life Sciences, Fujian Normal University, Qishan Campus, No.13 Science and Engineering Building, Fuzhou, Fujian 350117, China; ^5^The First Affiliated Hospital of Fujian Medical University, No.20 Chazhong Road, Fuzhou 350005, China; ^6^Affiliated Fuzhou Second Hospital of Xiamen University, No.47 Shangteng Road, Fuzhou 350007, China

## Abstract

**Background:**

Chlorogenic acid (CGA) is a polyphenolic compound with antioxidant and anti-inflammatory properties. CGA has been shown to improve neuroinflammation. This study is aimed at elucidating the exact mechanism by which CGA reduces neuroinflammation.

**Methods:**

Oxygen and glucose deprivation (OGD) was utilized to treat BV2 microglia and HT-22 hippocampal neurons to engineer an *in vitro* model of hypoxic ischemia reperfusion. The levels of inflammatory factors (IL-1*β*, IL-6, TNF-*α*, IL-4, and IL-10) and oxidative stress factors (MDA, SOD, and GSH-PX) in microglia were determined by ELISA kits. The neuron proliferation was assessed by CCK-8 assay, and LDH kit was used to determine LDH release in neurons. The fluorescent dye DCF-DA was employed to measure ROS levels in neurons. Correlation of MIR497HG, miR-29b-3p, and SIRT1/NF-*κ*B in neurons and microglia was determined by qRT-PCR. Expressions of inflammatory proteins (COX2, iNOS), oxidative stress pathways (Nrf2, HO-1), and apoptosis-related proteins (Bcl-2, Bax, caspase3, caspase8, and caspase9) in microglia or neurons were determined by western blot. The interactions between MIR497HG and miR-29b-3p, as well as between miR-29b-3p and SIRT1, were determined by dual luciferase assay and RIP assay.

**Results:**

CGA attenuated OGD-mediated inflammation and oxidative stress in microglia and inhibited microglia-mediated neuronal apoptosis. CGA increased the levels of MIR497HG and SIRT1 and suppressed the levels of miR-29b-3p in BV2 and HT-22 cells. MIR497HG knockdown, miR-29b-3p upregulation, and SIRT1 inhibition inhibited CGA-mediated anti-inflammatory and neuronal protective functions. There is a targeting correlation between MIR497HG, miR-29b-3p, and Sirt1. MIR497HG sponges miR-29b-3p to regulate SIRT1 expression in an indirect manner.

**Conclusion:**

CGA upregulates MIR497HG to curb miR-29b-3p expression, hence initiating the SIRT1/NF-*κ*B signaling pathway and repressing OGD-elicited inflammation, oxidative stress, and neuron apoptosis.

## 1. Introduction

Cerebral hypoxic ischemia (HI), the primary underlying pathogenesis of stroke and other neurological diseases, can contribute to severe neuron injury or death [1]. Destroyed redox homeostasis and neuroinflammation are crucial mechanisms resulting in hypoxic ischemia reperfusion brain tissue damage and neuron apoptosis [2]. Several studies have denoted that suppressing oxidative stress resulting from hypoxic ischemia reperfusion will be conducive to attenuating neuroinflammation and boosting neuron survival [3, 4]. Despite the huge progress made in the cellular and molecular pathogenesis of hypoxic ischemia reperfusion damage, we are still short of efficacious treatment strategies for hypoxic ischemia reperfusion patients. Thus, it is of great significance to seek novel methods for treating hypoxic ischemia reperfusion damage.

Chlorogenic acid (CGA, 3-CQA), a most abundant isomer among caffeoylquinic acid isomers (3-, 4-, and 5-CQA), carries various significant therapeutic functions like anti-inflammation, antioxidation, cardiac protection, anti-inflammation, antipyresis, and neuronal protection [5]. For instance, in the mouse ulcerative colitis model induced by dextran sulfate, CGA can impede the MAPK/ERK/JNK signaling pathway to substantially abate inflammation, oxidative stress, and cell apoptosis in colon tissues [6]. CGA can activate the Nrf2/HO-1 signaling pathway and hinder the NF-*κ*B pathway to dampen antioxidant and anti-inflammatory functions, thus guarding against diabetic nephropathy [7]. More of note, in the rat ischemic stroke model elicited by middle cerebral artery occlusion (MCAO), CGA lessens the generation of inflammatory factors and oxidative stress in the cerebral cortex of MCAO rats [8]. Notwithstanding, we are still in the dark about the function of CGA in hypoxic ischemia reperfusion-elicited brain damage.

Sirtuin-1 (SIRT1), a class III histone deacetylase (HDAC) and NAD^+^-dependent enzyme, deeply participates in gene regulation, maintenance of genomic stability, apoptosis, autophagy, senescence, proliferation, and tumorigenesis [9]. Recently, plentiful studies have disclosed that SIRT1 exerts a protective function in neuroinflammation-associated diseases [10]. For instance, in the OGD/R-elicited HT-22 neuron ischemia reperfusion model, the profile of SIRT1 is vigorously lowered, and SIRT1 upregulation considerably heightens HT-22 cell viability and lessens oxidative stress and neuron apoptosis [11]. Resveratrol initiates the SIRT1/NF-*κ*B signaling pathway in HI mice to mitigate HI-triggered long-term cognitive and memory deficits, hence attenuating neuroinflammatory responses. Based on the above findings, we can know that SIRT1 upregulation can ameliorate nerve damage induced by HI. In accordance with classical theories, lncRNAs can serve as the sponges of miRNAs, lowering their regulatory effects on mRNAs. For instance, in cerebral microvascular endothelial cells induced by OGD, lncRNA MALAT1 combines with miR-200c-3p and drives up SIRT1 expression to activate autophagy and bolster cell survival. Nonetheless, it remains poorly understood whether CGA can hamper hypoxic ischemia reperfusion-elicited nerve damage via the MIR497HG/miR-29b-3p/Sirt1 axis.

Here, we examined the impact of CGA on OGD-mediated microglia inflammation and neuron apoptosis and discovered that they could be dampened by CGA concentration dependently. Moreover, CGA uplifted the profiles of MIR497HG and SIRT1 and restricted the profile of miR-29b-3p in the cells. Therefore, we conjectured that CGA could upregulate MIR497HG and curb miR-29b-3p expression to initiate the Sirt1/NF-*κ*B signaling pathway and repress OGD-elicited inflammation, oxidative stress, and neuron apoptosis.

## 2. Materials and Methods

### 2.1. Cell Culture and Treatment

Mouse microglia (BV2), mouse hippocampal neurons (HT-22), and human embryonic kidney cells (HEK293T), ordered from the Shanghai Cell Bank of the Chinese Academy of Sciences (Shanghai, China), were cultured in a DMEM medium (Thermo Fisher HyClone, Utah, USA) supplemented with 5% FBS in an incubator with 5% CO_2_ at 37°C. The solution was renewed every two days, and the cells were passed every five days. We conducted the experiment as the cells grew to approximately 90% of the bottle bottom. BV2 and HT-22 cells were treated with CGA (5, 10, and 20 *μ*mol/L) for 24 hours beforehand and then with OGD for 6 hours. We prepared the conditioned medium (CM) of microglia: BV2 cells were pretreated with CGA of different concentrations for 24 hours and then exposed to OGD for 6 hours. The conditioned medium was obtained from the supernatant of BV2 cells subjected to OGD and treated with or without CGA. The MCM was harvested and administered to the HT-22 culture for 24-hour culture.

### 2.2. Cell Transfection

The pcDNA empty vector (NC, 5 *μ*g/mL), pcDNA-MIR497HG (MIR497HG, 5 *μ*g/mL), siRNA normal control (si-NC, 50 nM), siRNAs against MIR497HG (si-MIR497HG, 50 nM), miRNA control (miR-NC, 50 nM), miR-29b-3p mimics (miR-29b-3p, 50 nM), and miR-29b-3p inhibitors (miR-in, 100 nM) were supplied by GenePharma Co., Ltd. (Shanghai, China). BV2 and HT-22 cells, inoculated into 24-well plates with a density of 3 × 10^5^ cells/well, were incubated with 5% CO_2_ at 37°C for 24 hours and then subjected to cell transfection. Lipofectamine® 3000 (Invitrogen; Thermo Fisher Scientific, Inc.) was taken to transfect the above substances into BV2 and HT-22 cells as per the supplier's instructions. qRT-PCR confirmed the transfection efficiency. The cells were incubated with 5% CO_2_ at 37°C for 24 hours in preparation for further analysis. Following 24 hours' transfection, CGA and OGD were adopted to treat BV2 and HT-22 cells [12].

### 2.3. The Construction of the OGD Cell Model

We conducted OGD as described before [13]. Put simply, BV2 and HT-22 cells were cultured under hypoxic conditions (5% CO_2_, 0.2% O_2_) in a glucose-free medium for 6 hours. The plates were taken out from the anaerobic chamber, with the OGD medium substituted by a complete growth medium for 24 hours' further culture. The cells without being treated with OGD were taken as the control group. Following OGD, we harvested the supernatant and extracts of the cells for the following procedures.

### 2.4. Cell Viability Analysis

As instructed by the manufacturer, Cell Counting Kit-8 (CCK-8, Beyotime Institute of Biotechnology, Shanghai, China) was adopted to check cell viability. HT-22 neurons (5 × 10^4^ cells/well) were seeded into 96-well plates. After being incubated for 24 hours, the cells were administered with CGA (5, 10, and 20 *μ*M) and then subjected to OGD. Twenty-four hours later, 10 *μ*L CCK-8 was given to each well for 4 hours' further culture. A microplate reader (Bio-Rad, USA) was harnessed to gauge the absorbance value at 450 nm [14].

### 2.5. Determination of Lactate Dehydrogenase (LDH) Release

The LDH kit (Nanjing Jiancheng, China) was taken to determine LDH activity in the cell supernatant for evaluating HT-22 neuron damage [15]. After the neuron culture was exposed to OGD for 24 hours, the 100 *μ*L medium sucked out of each cell was transferred to 96-well plates and then incubated along with 100 *μ*L reaction mixture at room temperature (RT) for 10 minutes in darkness. We measured the optical density at 490 nm to confirm the amount of LDH release.

### 2.6. ELISA

BV2 cells induced by OGD were inoculated into 6-well plates, with 4 wells replicated in each group. Subsequent to 48 hours' culture, the cell supernatant was harvested and centrifuged at 1000 × *g* (4°C) for 10 minutes, and we obtained the wanted supernatant. The ELISA kits for interleukin-1*β* (IL-1*β*), interleukin-6 (IL-6), and tumor necrosis factor-*α* (TNF-*α*) were utilized to measure the contents of IL-1*β*, IL-6, and TNF-*α* in BV2 cells, respectively, strictly in line with the supplier's instructions.

### 2.7. Detection of Oxidative Stress Substances

The supernatant of BV2 cells elicited by OGD was harvested. The chemical colorimetric assay kit (Nanjing Jiancheng Bioengineering Institute) was adopted to check the concentration of malonaldehyde (MDA; cat. no. A003-4-1) and the activities of superoxide dismutase (SOD; cat. no. A001-3-2) and glutathione peroxidase (GSH-PX; cat. no. A005-1-2) in BV2 cells as per the manufacturer's instructions.

### 2.8. Determination of ROS in Cells

DCFH-DA was taken to examine reactive oxygen species (ROS) [16]. In brief, we incubated the neurons along with DCFH-DA for 30 minutes. The cells were flushed in PBS three times, and then, a fluorescence microscope was operated to gauge their fluorescence intensity at 488 nm.

### 2.9. Western Blot

Cell intervention in each group was implemented as mentioned before. The culture medium was removed, and the cells were flushed with PBS once. RIPA lysis buffer (Beyotime Biotechnology, Shanghai, China) supplemented with 1% phenylmethylsulfonyl fluoride (PMSF) was adopted to extract proteins out of the cells, with the protein content measured through the BCA method. Following protein denaturation, the proteins were separated through 10% SDS-PAGE gel electrophoresis and then moved onto polyvinylidene fluoride (PVDF) membranes (Millipore, Bedford, MA, USA) at a constant current of 300 mA. After being sealed with 5% skimmed milk powder for an hour, the membranes were incubated along with primary antibodies anti-COX2 (Abcam, 1 : 1000, ab179800, MA, USA), anti-iNOS (1 : 1000, ab178945), anti-SIRT1 (1 : 1000, ab189494), anti-Nrf2 (1 : 1000, ab137550), anti-HO-1 (1 : 1000, ab52947), anti-NF-*κ*B (1 : 1000, ab32536), anti-pNF-*κ*B (1 : 1000, ab76302), anti-Bcl-2 (1 : 1000, ab32124), anti-Bax (1 : 1000, ab32503), anti-cleaved-caspase3 (1 : 1000, ab32042), anti-cleaved-caspase8 (Art. No. PA5-99435, Thermo Fisher, USA), anti-cleaved-caspase9 (1 : 1000, ab2324), and anti-*β*-actin (1 : 1000, ab6276) overnight at 4°C. Following a routine wash, the membranes were incubated along with the secondary antibody at RT for 60 minutes and then rinsed with TBST 4 times, 8 minutes each. The Pierce ECL Western Blot Substrate Kit (Amersham Pharmacia Biotech, Little Chalfont, UK) supplied by Thermo was introduced for X-ray development.

### 2.10. Quantitative Reverse Transcription Polymerase Chain Reaction (RT-qPCR)

TRIzol reagent (Invitrogen, Carlsbad, CA, USA) was adopted to extract lncRNAs and miRNAs out of BV2 microglia and HT-22 neurons. The PrimeScript® RT reagent kit (TaKaRa, Dalian, Liaoning, China) and the MicroRNA Reverse Transcription kit (Takara, Shiga, Japan) were employed to reverse transcribe the lncRNAs and miRNAs into cDNAs, respectively. Next, real-time fluorescence quantitative PCR was implemented with the use of SYBR Green PCR reagent and ABI7500FAST Real-Time PCR. The 2^-*ΔΔ*Ct^ method was introduced to assess the profiles of MIR497HG and miR-29b-3p. GAPDH was taken as the internal parameter of MIR497HG, and U6 was regarded as that of miR-29b-3p. MIR497HG: forward: 5′-ATAAGAATCCAGGTCGGGGC-3′, reverse: 5′-CCCAAGGTTCCATCGTCCTC-3′; miR-29b-3p: forward: 5′-GGGGGTACCCTTCAGGAAGCTGGTTTC-3′, reverse: 5′-GGGGATATCTACATGTGAGGCAGGTTCTCAC-3′; GAPDH: forward: 5′-GAAGATGGTGATGGGATTTC-3′, reverse: 5′-GAAGGTGAAGGTCGGAGT-3′; U6: forward: 5′-CTCGCTTCGGCAGCACA-3′, reverse: 5′-AACGCTTCACGAATTTGCGT-3′.

### 2.11. Dual Luciferase Reporter Gene Assay

Lipofectamine 2000 transfection reagent (Invitrogen) was adopted to transfect the Wt (Mut) MIR497HG vector or the Wt (Mut) 3′UTR of the SIRT1 vector and miR-29b-3p mimics or simulated NC into HEK293T cells. The dual luciferase assay system (Ambion, Austin, TX, USA) was exploited to examine the cells' luciferase activity following 48 hours' transfection [17].

### 2.12. RNA Immunoprecipitation (RIP) Assay

The correlations between lncRNA MIR497HG and miR-29b-3p, as well as between miR-29b-3p and SIRT1, were confirmed through the Magna RIP RNA binding protein immunoprecipitation kit (Millipore, USA) [18]. In brief, BV2 cells (2 × 10^7^) or HT-22 cell lysates were incubated along with magnetic beads conjugated with the negative control normal mouse IgG or the human anti-Ago2 antibody (Millipore). qRT-PCR examined the profiles of MIR497HG and miR-29b-3p in the lysates.

### 2.13. Statistical Analysis

The SPSS 21.0 statistical software (SPSS Inc., Chicago, IL, USA) was introduced for statistical analysis, with the measurement statistics presented as mean ± standard deviation (*X* ± *S*). One-way ANOVA was carried out to analyze the measurement data. Each independent experiment was conducted three times. An independent sample *t*-test was taken for comparison between groups. *P* < 0.05 was regarded as statistically meaningful.

## 3. Results

### 3.1. Chlorogenic Acid Hampered Inflammation and Oxidative Stress in Microglia Induced by OGD

To confirm whether CGA treatment was correlated with inhibition of proinflammatory mediator and oxidative stress substance secretion, we treated BV2 cells beforehand with CGA (5-20 *μ*M) for 24 hours and then treated them with OGD for 6 hours. It turned out that in contrast with the Con group, there was an increase in the levels of IL-1*β*, IL-6, and TNF-*α* and a reduction in those of IL-4 and IL-10 in BV2 cells elicited by OGD. CGA substantially curbed the levels of IL-1*β*, IL-6, and TNF-*α* and augmented those of IL-4 and IL-10 in a dose-dependent pattern (Figure 1(a)). Commercial kits were utilized to examine the levels of MDA, SOD, and GSH-PX in OGD-elicited BV2 cells. As a result, by contrast to the Con group, the level of MDA was heightened, while the activities of SOD and GSH-PX were notably lowered in the induced cells, but CGA contributed to the opposite situation (Figure 1(b)). Moreover, western blot measured the profiles of inflammatory proteins (COX2, iNOS) and antioxidative stress proteins (Nrf2, HO-1) in BV2 cells induced by OGD. It displayed that in contrast with the Con group, the protein levels of COX2 and iNOS were heightened, and those of Nrf2 and HO-1 remained the same. CGA considerably suppressed the profiles of COX2 and iNOS and further augmented the profiles of Nrf2 and HO-1 in OGD-elicited BV2 cells (Figures 1(c) and 1(d)). All these findings revealed that CGA repressed OGD-mediated inflammation and oxidative stress in microglia.

### 3.2. Chlorogenic Acid Impeded Neuron Apoptosis and Oxidative Stress Mediated by OGD

To investigate the impact of CGA on neurons, we treated HT-22 cells with CGA (5-20 *μ*M) for 24 hours and then exposed them to OGD for 6 hours. As evidenced by CCK-8, in contrast with the Con group, neuron apoptosis induced by OGD was dramatically expanded, whereas CGA dose dependently cramped it (Figure 2(a)). Western blot revealed that by contrast to the Con group, the profiles of proapoptotic proteins Bax, C-caspase3, C-caspase8, and C-caspase9 were remarkably uplifted, but the profile of the antiapoptotic protein Bcl-2 was substantially lessened in the induced neurons. In contrast with the OGD group, CGA considerably suppressed the protein profiles of Bax, C-caspase3, C-caspase8, and C-caspase9 and augmented Bcl-2 protein expression in a dose-dependent manner (Figure 2(b)). To assess whether CGA could guard against oxidative stress elicited by OGD, we determined ROS levels in HT-22 cells and discovered that ROS levels were distinctly higher in the OGD group than in the Con group. CGA conspicuously brought down ROS levels in the cells elicited by OGD (Figure 2(c)). The LDH kit was harnessed to monitor LDH release in OGD-elicited HT-22 cells, indicating that LDH release was substantially higher in the OGD group than in the Con group, whereas the level of LDH was greatly lowered by CGA (Figure 2(d)). All our outcomes demonstrated that CGA hampered OGD-mediated neuron apoptosis and oxidative stress.

### 3.3. Chlorogenic Acid Curbed Neuron Apoptosis Mediated by Microglia

To ascertain the influence of microglia on neurons, we harvested the conditioned medium of microglia and administered it to HT-22 cells for 24 hours' incubation. Later on, we confirmed CGA's potential in neuroprotection by checking HT-22 cell viability through CCK-8 and by examining apoptosis-concerned proteins via western blot to evaluate cell apoptosis. The figures displayed that in contrast with the CM^con^ group, the conditioned medium of activated microglia triggered a reduction in HT-22 cell viability, but CGA (20 *μ*M) vigorously bolstered the cells' survival and curbed their apoptosis (Figures 3(a) and 3(b)). We also tested ROS levels and LDH release in HT-22 cells and uncovered that as opposed to the CM^con^ group, the CM^OGD^ group witnessed a distinct rise in the levels of ROS and LDH. CGA (20 *μ*M) vigorously dampened their levels in the CM^OGD^ group (Figures 3(c) and 3(d)). All these phenomena denoted that microglia induced by OGD could foster neuron damage, whereas CGA could hinder neuron apoptosis mediated by microglia.

### 3.4. Chlorogenic Acid Upregulated MIR497HG and SIRT1 and Restrained miR-29b-3p

To verify whether MIR497HG was indispensable to inflammation elicited by OGD and whether CGA's inhibitory impact on neuroinflammatory responses was associated with its regulation on MIR497HG, we measured the profiles of MIR497HG, miR-29b-3p, and SIRT1 in OGD-induced BV2 and HT-22 cells via qRT-PCR and western blot. As a result, in contrast with the Con group, there was a decline in the profiles of MIR497HG, SIRT1, and pNF-*κ*B and a rise in miR-29b-3p expression in the induced cells, whereas CGA dose dependently uplifted the profiles of MIR497HG, SIRT1, and pNF-*κ*B and restrained miR-29b-3p expression (Figures 4(a)–4(f)). The above findings disclosed that CGA could dose dependently heighten the profiles of MIR497HG and SIRT1 and restricted miR-29b-3p expression in OGD-elicited cells.

### 3.5. miR-29b-3p Was Targeted by MIR497HG and Targeted SIRT1

The bioinformatics prediction database was utilized to analyze the downstream targets of MIR497HG and miR-29b-3p. It transpired that binding sites existed between MIR497HG and miR-29b-3p and between miR-29b-3p and SIRT1 (Figure 5(a)). To ascertain the interplay between MIR497HG and miR-29b-3p, as well as between miR-29b-3p and SIRT1, we conducted dual luciferase assay. The outcomes exhibited that following the transfection of miR-29b-3p mimics, the relative luciferase activities of MIR497HG-WT and STAT1-WT were apparently lowered in HEK293T cells, but the activities of the mutant vectors remained the same (Figures 5(b) and 5(c)). RIP further determined their correlations. By contrast to the control IgG, MIR497HG and miR-29b-3p were preferentially enriched in the beads incorporating Ago2, which indicated that miR-29b-3p was the miRNA targeted by MIR497HG (Figure 5(d)). At last, qRT-PCR and western blot were carried out to gauge the profiles of miR-29b-3p and SIRT1 in BV2 and HT-22 cells following overexpression of MIR497HG or miR-29b-3p. As a result, in contrast with the vector group, MIR497HG overexpression contributed to a stark decline in miR-29b-3p expression and a distinct increase in SIRT1 expression, whereas MIR497HG inhibition resulted in the opposite consequences. In contrast with the miR-NC group or the miR-in group, miR-29b-3p upregulation or downregulation could dampen or augment SIRT1 expression (Figures 5(e)–5(h)). These outcomes revealed that miR-29b-3p was targeted by MIR497HG and targeted SIRT1.

### 3.6. MIR497HG Knockdown Inverted Chlorogenic Acid-Mediated Anti-Inflammatory and Neuroprotective Functions

To confirm whether MIR497HG participated in the process of CGA exerting its neuroprotective effect, we transfected Si-NC and Si-MIR497HG into BV2 and HT-22 cells and treated them with CGA (20 *μ*M) and OGD 24 hours later. ELISA and western blot revealed that in contrast with the OGD+CGA group, MIR497HG inhibition elevated the profiles of inflammatory factors and inflammatory proteins in BV2 cells (Figures 6(a) and 6(b)), facilitated the generation of oxidative stress factors, and repressed the profiles of antioxidative stress proteins (Figures 6(c) and 6(d)). Moreover, CCK-8 and western blot denoted that in contrast with the OGD+CGA group, MIR497HG inhibition suppressed neuron proliferation, boosted neuron apoptosis (Figures 6(e) and 6(f)), and bolstered ROS production (Figure 6(g)) and LDH release (Figure 6(h)) in neurons. The above findings unraveled that MIR497HG knockdown upended chlorogenic acid-mediated anti-inflammatory and neuroprotective functions.

### 3.7. miR-29b-3p Overexpression Inverted Chlorogenic Acid-Mediated Anti-Inflammatory and Neuroprotective Functions

To understand the influence of miR-29b-3p on CGA, we transfected miR-NC and miR-29b-3p mimics into BV2 and HT-22 cells. Twenty-four hours later, CGA (20 *μ*M) and OGD were adopted to treat BV2 and HT-22 cells. In contrast with the OGD+CGA group, miR-29b-3p upregulation augmented inflammation and oxidative stress in BV2 cells, suppressed the profiles of antioxidative stress proteins in the cells (Figures 7(a)–7(d)), enhanced neuron apoptosis (Figures 7(e) and 7(f)), and uplifted ROS levels (Figure 7(g)) and LDH release (Figure 7(h)) in neurons. These outcomes unveiled that miR-29b-3p upended the anti-inflammatory and neuroprotective effects mediated by chlorogenic acid.

### 3.8. SIRT1 Inhibition Counteracted the Anti-Inflammatory and Neuroprotective Functions Mediated by Chlorogenic Acid

The above discoveries exhibited that CGA could dose dependently elevate SIRT1 expression in OGD-elicited cells. Next, BV2 and HT-22 cells were treated with the SIRT1 inhibitor EX527 (50 *μ*M) in the presence or absence of CGA and then subjected to OGD treatment. In contrast with the OGD+CGA group, SIRT1 inhibition conspicuously inverted the anti-inflammatory and neuroprotective functions mediated by CGA: inflammation and oxidative stress were enhanced in BV2 cells (Figures 8(a)–8(c)), the profiles of antioxidative stress proteins were lessened (Figure 8(d)), neuron apoptosis was facilitated (Figures 8(e) and 8(f)), and the profile of ROS (Figure 8(g)) and the release of LDH (Figure 8(h)) were boosted in neurons. All these discoveries unraveled that SIRT1 inhibition upended chlorogenic acid-mediated anti-inflammatory and neuroprotective functions.

## 4. Discussion

Long noncoding RNAs (lncRNAs), novel noncoding RNAs with a length of over 200 nucleotides, play an essential part in inflammatory responses and diseases [19]. Reportedly, hypoxia and ischemia in the aftermath of lessened or interrupted cerebral blood flow can bring about alterations in the profiles of many lncRNAs in brain tissues, hence influencing disease progression [20–23]. lncRNA MIR497HG (MIR497HG), a member of the lncRNA family, targets the miRNA-128-3p/SIRT1 axis to suppress proliferation and migration in human retinal endothelial cells elicited by high glucose [24]. Nevertheless, the function of MIR497HG in hypoxic ischemia reperfusion-caused brain damage remains obscure.

MicroRNAs (miRNAs), small noncoding RNAs, can repress messenger RNA (mRNA) translation or facilitate mRNA degradation to modulate gene expression after transcription [25]. microRNA-29b-3p (miR-29b-3p), a member of the miRNA family, is believed to boast proinflammatory activities in inflammatory diseases like chronic respiratory diseases [26], sepsis-induced myocardial damage [27], osteoarthritis [28], and nephritis [29]. miR-29b-3p expression inhibition can cramp inflammatory factor production. On the other side of the fence, miR-29b-3p expression is greatly uplifted in the serum of ischemic stroke patients [30], but its exact role is rarely investigated. Thus, we probed into the profile and function of miR-29b-3p in the *in vivo* and *in vitro*hypoxic ischemia reperfusion models here.

Hypoxic-ischemic injury is not only the primary pathogenesis of cerebrovascular diseases like stroke and neurodegenerative diseases but also a leading contributor to the morbidity and mortality of newborns [31]. Once neurons are deprived of oxygen or blood supply, umpteen pathological events will be triggered, including oxidative stress, inflammation, and apoptosis, and neurodegeneration will also follow [32]. Microglia, resident immune cells in the central nervous system, exert a critical function in inflammatory responses in the brain [33, 34]. Suppressing inflammation and oxidative stress in microglia can mitigate brain damage induced by hypoxia-ischemia [35, 36]. Therefore, anti-inflammatory or antioxidant reagents are extremely promising in preventing or ameliorating neuron damage in the wake of ischemia-reperfusion. CGA, a potent natural antioxidant, is of great significance in kidney damage [37] and myocardial infarction [38] thanks to its anti-inflammatory and antioxidant functions. Here, we concentrated on the neuroprotective function of CGA in the context of cerebral hypoxia and ischemia.

Under various pathological conditions, chlorogenic acid boasts specific anti-inflammatory and antioxidant functions [39]. For instance, CGA may attenuate proinflammatory and apoptotic mediators and boost the antioxidant ability of liver tissues, thus eliminating liver toxicity induced by methotrexate (MTX) [40]. More of note, apple phenolic extracts (APEs) containing CGA can treat lead-caused neurotoxicity and neurodegenerative diseases through their antioxidant, anti-inflammatory, and antiapoptotic effects [41]. Here, we discovered that after intervening in BV2 and HT-22 cells for 24 hours beforehand, CGA dose dependently abated inflammatory and oxidative responses in BV2 cells induced by OGD and impeded neuron apoptosis.

Prior works have disclosed that many lncRNAs mediate hypoxic-ischemic brain damage progression, including MALAT1 [42], KCNQ1OT1 [43], lncRNA NEAT1 [44], and lncRNA GAS5 [45]. MIR497HG is a member of the lncRNA family, but the current studies on it mostly concentrate on tumors [46, 47], while its role in neuroinflammation has not been probed. A valuable discovery is that MIR497HG is an underlying relevant lncRNA in the context of ischemic stroke, but its function in the disease has not yet been investigated [48]. Here, we corroborated that the level of MIR497HG was substantially lowered in OGD-elicited BV2 cells and neurons, whereas CGA could heighten its profile in cells. MIR497HG knockdown reversed the anti-inflammatory and neuroprotective effects mediated by chlorogenic acid.

Increasing evidence has substantiated that miRNAs are indispensable to the occurrence and progression of hypoxic ischemia reperfusion brain damage. For instance, miR-3473b expression is uplifted in the cortex and striatum of MCAO mice. The intraventricular injection of miR-3473b antagomir prior to MCAO vigorously weakens the profiles of miR-3473b and proinflammatory factors induced by ischemia in the brain tissues of MCAO mice and lessens the infarction area of the mice post-MCAO [49]. miR-181c can directly target the 3′-untranslated region of TNF-*α* mRNA, alleviate inflammation in OGD-elicited microglia, and hamper neuron apoptosis mediated by microglia [50]. Moreover, other miRNAs like miR-26b [51], miR-455-3p [52], miR-199a-5p [53], and miR-142-3p [54] also partake in hypoxic-ischemic brain injury development. miR-29b-3p can modulate inflammation in diseases like chronic respiratory disease [26], sepsis-induced myocardial damage [27], and osteoarthritis [28], and miR-29b-3p mimics can weaken the anti-inflammatory function of BMSC exosome H19 in BV2 cells stimulated by LPS in the context of neuroinflammatory diseases [55]. Nevertheless, the role of miR-29b-3p in hypoxic-ischemic brain damage has not been discovered [56]. Here, we uncovered that CGA could dampen the profile of miR-29b-3p in OGD-induced BV2 cells and neurons. miR-29b-3p upregulation inverted chlorogenic acid-mediated anti-inflammatory and neuroprotective effects.

SIRT1, the most outstanding and most extensively investigated member among Sirtuins, is known as a nuclear protein that regulates biological processes like inflammation, oxidative stress, mitochondrial function, immune response, cell differentiation, proliferation, and metabolism [57]. SIRT1 signaling pathway activation can suppress inflammatory cytokines and cell apoptosis to modulate brain damage incurred by ischemic stroke [58]. For instance, resveratrol can initiate SIRT1 so as to influence the deacetylation and nuclear translocation of the nuclear factor-kappa B (NF-*κ*B) subunit p65, hence alleviating neuroinflammation mediated by the NF-*κ*B axis as well as hippocampal neuron injury [59]. Our research also attained the same outcomes. CGA could augment the profile of SIRT1/NF-*κ*B in OGD-elicited BV2 cells and HT-22 neurons, and SIRT1 inhibition inverted the anti-inflammatory and neuroprotective functions mediated by chlorogenic acid. It is widely understood that lncRNAs can serve as the sponges of miRNAs and thus lower their regulatory impact on mRNAs. Bioinformatics analysis confirmed that there were binding sites between MIR497HG and miR-29b-3p, as well as between miR-29b-3p and SIRT1. Dual luciferase assay and RIP corroborated the targeted binding correlations between MIR497HG and miR-29b-3p and between miR-29b-3p and SIRT1. We also demonstrated that CGA could upregulate MIR497HG, target and repress miR-29b-3p expression, and upregulate SIRT1 to lessen inflammation in OGD-elicited BV2 cells and curb HT-22 neuron apoptosis following OGD stimulation.

All in all, we have demonstrated that CGA can dose dependently hamper neuroinflammation and abate neuron apoptosis. CGA heightens MIR497HG and SIRT1 expressions and restrains miR-29b-3p expression. Moreover, MIR497HG and SIRT1 inhibition or miR-29b-3p upregulation can upend the anti-inflammatory and neuroprotective functions of CGA. All these discoveries display that CGA can modulate the MIR497HG-miR-29b-3p-SIRT1 axis (Supplementary Figure 1) and can be utilized as a novel treatment strategy for hypoxic ischemia reperfusion brain damage.

## Figures and Tables

**Figure 1:** Chlorogenic acid repressed inflammation and oxidative stress in OGD-elicited microglia. CGA (5-20 *μ*M) was adopted to treat BV2 cells for 24 hours, which were then exposed to OGD for 6 hours. (a) ELISA examined the profiles of IL-6, IL-1*β*, TNF-*α*, IL-4, and IL-10 in BV2 cells. (b) Western blot confirmed the protein profiles of COX2 and iNOS in BV2 cells. (c) Commercial kits were taken to check the profiles of MDA, SOD, and GSH-PX in BV2 cells. (d) Western blot determined the protein profiles of Nrf2 and HO-1 in BV2 cells. Statistics were presented as mean ± SD. *N* = 3. NS *P* > 0.05, ^∗∗^*P* < 0.01, and ^∗∗∗^*P* < 0.001 (vs. the Con group). ^&^*P* < 0.05, ^&&^*P* < 0.01, and ^&&&^*P* < 0.001 (vs. the OGD group).

**Figure 2:** Chlorogenic acid curbed neuron apoptosis and oxidative stress mediated by OGD. To confirm the influence of CGA on neurons, we treated HT-22 cells with the use of CGA (5-20 *μ*M) for 24 hours and then exposed them to OGD for 6 hours. (a) CCK-8 examined cell proliferation. (b) Western blot confirmed the protein profiles of Bax, C-caspase3, C-caspase8, C-caspase9, and Bcl-2 in cells. (c) Confocal microscopy images exhibited the immunofluorescence staining of ROS in HT-22 cells. Scale = 100 *μ*m. (d) The LDH kit was adopted to monitor LDH release in cells. Statistics were presented as mean ± SD. *N* = 3. NS *P* > 0.05, ^∗∗^*P* < 0.01, and ^∗∗∗^*P* < 0.001 (vs. the Con group). ^&^*P* < 0.05, ^&&^*P* < 0.01, and ^&&&^*P* < 0.001 (vs. the OGD group).

**Figure 3:** Chlorogenic acid suppressed neuron apoptosis mediated by microglia. The conditioned medium of microglia was harvested and administered to HT-22 cells for 24 hours' incubation. (a) CCK-8 examined cell proliferation. (b) Western blot confirmed the protein profiles of Bax, C-caspase3, C-caspase8, C-caspase9, and Bcl-2 in cells. (c) Confocal microscopy images displayed the immunofluorescence staining of ROS in HT-22 cells. Scale = 100 *μ*m. (d) The LDH kit was taken to monitor LDH release in cells. Statistics were presented as mean ± SD. *N* = 3. NS *P* > 0.05, ^∗∗^*P* < 0.01, and ^∗∗∗^*P* < 0.001 (vs. the CM^con^ group). ^&&^*P* < 0.01 and ^&&&^*P* < 0.001 (vs. the CM^OGD^ group).

**Figure 4:** Chlorogenic acid upregulated MIR497HG and SIRT1 and cramped miR-29b-3p. (a, b) qRT-PCR examined the profiles of MIR497HG and miR-29b-3p in BV2 cells that were treated in the presence or absence of CGA (5-20 *μ*M) and induced by OGD. (c) Western blot confirmed the profiles of SIRT1 and pNF-*κ*B in the BV2 cells. (d, e) qRT-PCR determined the profiles of MIR497HG and miR-29b-3p in HT-22 cells treated in the presence or absence of CGA (5-20 *μ*M) and induced by OGD. (f) Western blot checked the profiles of SIRT1 and pNF-*κ*B in the HT-22 cells. Statistics were presented as mean ± SD. *N* = 3. ^∗∗∗^*P* < 0.001 (vs. the Con group). ^&^*P* < 0.05, ^&&^*P* < 0.01, and ^&&&^*P* < 0.001 (vs. the OGD group).

**Figure 5:** miR-29b-3p was targeted by MIR497HG and targeted SIRT1. (a) The Starbase website forecast the binding sites between MIR497HG and miR-29b-3p, as well as between miR-29b-3p and SIRT1. (b, c) Dual luciferase reporter gene assay analyzed the luciferase activity of HEK-293T cells transfected together with miR-29b-3p mimics, MIR497HG-WT (or MIR497HG-MUT), and SIRT1-WT (or SIRT1-MUT). NS *P* > 0.05 and ^∗∗^*P* < 0.01 (vs. the miR-NC group). (d) RIP confirmed the binding correlation between MIR497HG and miR-29b-3p in cells. ^∗∗∗^*P* < 0.001 (vs. the IgG group). (e, f) qRT-qPCR gauged the profile of miR-29b-3p in BV2 and HT-22 cells after MIR497HG upregulation or downregulation. (g, h) Western blot checked the profiles of SIRT1 and pNF-*κ*B in BV2 and HT-22 cells following miR-29b-3p upregulation or downregulation. Statistics were presented as mean ± SD. *N* = 3. ^∗∗^*P* < 0.01 and ^∗∗∗^*P* < 0.001 (vs. the vector or miR-NC group). ^&&^*P* < 0.01 and ^&&&^*P* < 0.001 (vs. the si-NC or miR-in group).

**Figure 6:** MIR497HG knockdown inverted the anti-inflammatory and neuroprotective functions mediated by chlorogenic acid. BV2 and HT-22 cells were transfected along with Si-NC and Si-MIR497HG. Twenty-four hours later, CGA (20 *μ*M) and OGD were taken to treat the cells for 24 hours. (a) ELISA verified the profiles of IL-6, IL-1*β*, TNF-*α*, IL-4, and IL-10 in BV2 cells. (b) Western blot confirmed the protein profiles of COX2 and iNOS in BV2 cells. (c) Commercial kits were utilized to check the profiles of MDA, SOD, and GSH-PX in BV2 cells. (d) Western blot revealed the protein profiles of Nrf2 and HO-1 in BV2 cells. (e) CCK-8 monitored HT-22 cell proliferation. (f) Western blot ascertained the protein profiles of Bax, C-caspase3, C-caspase8, C-caspase9, and Bcl-2 in HT-22 cells. (g) Confocal microscopy images displayed the immunofluorescence staining of ROS in HT-22 cells. Scale = 100 *μ*m. (h) The LDH kit was adopted to monitor LDH release in cells. Statistics were presented as mean ± SD. *N* = 3. ^∗^*P* < 0.05, ^∗∗^*P* < 0.01, and ^∗∗∗^*P* < 0.001 (vs. the OGD+si-NC group). ^&&^*P* < 0.01 and ^&&&^*P* < 0.001 (vs. the OGD+CGA group).

**Figure 7:** miR-29b-3p overexpression inverted chlorogenic acid-mediated anti-inflammatory and neuroprotective functions. miR-NC and miR-29b-3p mimics were transfected into BV2 and HT-22 cells. Twenty-four hours later, CGA (20 *μ*M) and OGD were employed to treat the cells. (a) ELISA examined the profiles of IL-6, IL-1*β*, TNF-*α*, IL-4, and IL-10 in BV2 cells. (b) Western blot gauged the protein profiles of COX2 and iNOS in BV2 cells. (c) Commercial kits were utilized to check the profiles of MDA, SOD, and GSH-PX in BV2 cells. (d) Western blot revealed the protein profiles of Nrf2 and HO-1 in BV2 cells. (e) CCK-8 checked HT-22 cell proliferation. (f) Western blot ascertained the protein profiles of Bax, C-caspase3, C-caspase8, C-caspase9, and Bcl-2 in HT-22 cells. (g) Confocal microscopy images displayed the immunofluorescence staining of ROS in HT-22 cells. Scale = 100 *μ*m. (h) The LDH kit was harnessed to monitor LDH release in cells. Statistics were presented as mean ± SD. *N* = 3. ^∗^*P* < 0.05, ^∗∗^*P* < 0.01, and ^∗∗∗^*P* < 0.001 (vs. the OGD+miR-NC group). ^&^*P* < 0.05, ^&&^*P* < 0.01, and ^&&&^*P* < 0.001 (vs. the OGD+CGA group).

**Figure 8:** Inhibition of SIRT1 counteracted chlorogenic acid-mediated anti-inflammatory and neuroprotective effects. In the presence or absence of CGA, BV2 and HT-22 cells were treated with the SIRT1 inhibitor EX527 (50 *μ*M) and then exposed to OGD. (a) ELISA confirmed the profiles of IL-6, IL-1*β*, TNF-*α*, IL-4, and IL-10 in BV2 cells. (b) Western blot determined the protein profiles of COX2 and iNOS in BV2 cells. (c) Commercial kits were taken to measure the profiles of MDA, SOD, and GSH-PX in BV2 cells. (d) Western blot verified the protein profiles of Bax, C-caspase3, C-caspase8, C-caspase9, and Bcl-2 in HT-22 cells. (g) Confocal microscopy images exhibited the immunofluorescence staining of ROS in HT-22 cells. Scale = 100 *μ*m. (h) The LDH kit detected LDH release in cells. Statistics were presented as mean ± SD. *N* = 3. ^∗∗^*P* < 0.01 and ^∗∗∗^*P* < 0.001 (vs. the OGD+EX527 group). ^&&^*P* < 0.01 and ^&&&^*P* < 0.001 (vs. the OGD+CGA group).

## Data Availability

All data was included in our manuscript.

## Supplementary Materials

Supplementary Materials The correlation between MIR497HG, miR-29b-3p, and Sirt1.
